# Study on Key Drivers and Collaborative Management Strategies for Construction and Demolition Waste Utilization in New Urban District Development: From a Social Network Perspective

**DOI:** 10.1155/2023/3660647

**Published:** 2023-02-09

**Authors:** Ling Shen, Zhaokun Zhang, Lingyi Tang

**Affiliations:** ^1^Department of Construction Management, School of Civil Engineering, Sanjiang University, No. 310 Longxi Road Yuhuatai District, Nanjing, Jiangsu, China; ^2^Department of Smart Construction and Management, School of Civil Engineering, Nanjing Tech University, No. 30 Puzhu South Road Pukou District, Nanjing, Jiangsu, China; ^3^Department of Construction Management and Real Estate, School of Civil Engineering, Southeast University, Jiulonghu Campus Nanjing, Nanjing, Jiangsu, China

## Abstract

Construction and demolition waste (C&DW) during new district development shows the characteristics of large quantity, concentrated distribution, and long duration on both supply and demand sides. The construction of the new district has objective conditions to promote the scale development of recycling industries and achieve green development through local digestion, so the recycling indicators for the new district proposed by the government are generally higher than those of other regions. However, many new districts have yet to systematically identify key drivers (KDs) of recycling and form win-win governance mechanisms with multiple government and market subjects, resulting in uncontrolled accumulation or high-cost discard of C&DW. This paper identifies 29 recycling drivers and 8 governing subjects through literature research and a field study of five national new districts in China. Then, a 2-mode social network and two 1-mode social networks are constructed to analyze the complex interactions between drivers and governing subjects, taking Nanjing Jiangbei New District as an example. The results of the study show that most of the drivers need at least 2 governance subjects to promote together, which indicates that it is necessary to build a collaborative governance mechanism of multiple subjects. This study provides a structured framework to analyze the drivers of recycling in new district development and the collaborative governance of multiple subjects, which can provide a basis for promoting efficient recycling of new district development.

## 1. Introduction

Urban new districts, including national new districts and new districts set up by local governments, are one of the forms of high-quality and rapid urban development and expansion in the urbanization process [1]. There are 19 national-level new districts in China, with a total scale of more than 50,000 square kilometers, which have become an important growth pole for national and local economic and social sustainable development. During the development and construction of a new district, a large number of buildings and structures need to be demolished and constructed, thus generating a large amount of C & DW. At the same time, the development of the new district also provides a better platform for low-cost (large-scale disposal, production and sales, and short transportation distances) and high-efficiency utilization of C & DW. This is because of the large volume and concentrated distribution of C&DW generated in the construction of new districts, the long duration of new projects, the high positioning of construction standards and environmental requirements, and the need for a large amount of new construction materials. In addition, new projects with large volumes, long durations, and large construction can also provide sites for the construction of temporary fixed resource-based disposal facilities (on-site treatment facilities that can exist for 3 to 6 years), offering the possibility of building mobile disposal facilities, temporary fixed and long-term fixed disposal facilities that can develop in parallel with efficient resource-based disposal modes in new areas.

Based on the pressure and requirements of sustainable development, C&DW's recycling research is receiving attention not only in China, but also around the world. Many scholars have studied the drivers of recycling, emphasizing the need to explore a collaborative governance mechanism led by the government, operated by social capital, and participated by the public, and to use this collaborative effect to improve the level of recycling, so as to get out of the governance dilemma of C&DW [2–4]. However, few studies have systematically considered the interactions among the various drivers and the role of each governance subject on the drivers, leading to deviations between theoretical studies and actual situations. Moreover, there are no studies related to the multiple and complex relationships between recycling drivers and governance subjects that characterize the development of new districts.

In order to address the above issues, the following actions are critical: the first is to identify the drivers affecting the recycling of new district development and the collaborative governance subjects of the whole recycling process. Then, analyze the complex relationships among the drivers, the governance subjects, and between the drivers and the governance subjects. The advantage of SNA over other research methods is that it can provide quantitative metrics for analyzing the relationships between nodes in a network. Therefore, this paper proposes to study the abovementioned multiple complex relationships based on SNA to provide a framework for the analysis of the new district C&DW recycling. The results of the study can prompt multiple governance subjects to adopt effective strategies for efficient collaboration and quick linkage to achieve the new district C&DW recycling goal.

The remainder of the paper is organized as follows: the second section provides a detailed literature review of drivers and collaborative governance affecting C&DW recycling to identify knowledge gaps in the field. The third section describes the research methodology. In the fourth part, the SNA model is established using 29 drivers and 8 governance subjects identified from the literature study and the research of 5 national new districts in China as network nodes. The SNA method is used to analyze the drivers and the characteristic indicators of the 2-mode network of governance subjects to determine the role of different governance subjects in drivers and to verify the relationship between drivers and governance subjects. Then, the two 1-mode networks of drivers and governance subjects are analyzed to further reveal their internal relationships. Finally, a collaborative governance strategy is proposed according to the results of the SNA.

## 2. Literature Review

### 2.1. Literature on C&DW Recycling Drivers

Based on the fact that the attitudes and behaviors of owners and contractors at both the supply and demand ends of the C&DW reverse supply chain are the fundamental drivers of recycling, related research is conducted mainly from the perspective of owners and contractors. Jain et al. [5] propose that the behavioral choices of owners are mainly influenced by perceived benefits, perceived costs, attitudes, subjective norms and perceived behavioral control, institutional pressures, and environmental awareness. Al-Sari et al. [6] and Yu et al. [7], on the other hand, suggest that the factors influencing contractors' behavior in purchasing recycled products are mainly government measures, perceived behavioral control, perceived effectiveness, subjective norms, and the influence of recycled product information. In the absence of a regulatory framework, the voluntary attitudes and behaviors of contractors are driven primarily by direct economic considerations.

Early research on the environmental conditions required for recycling was mainly from a policy-making perspective. Jimenez–Rivero and Garcia–Navarro [8] pointed out that government regulatory instruments must be used in conjunction with economic instruments or other control strategies, emphasizing that policies as well as relevant laws and regulations are the KDs of recycling. Jia et al. [9] further used a system dynamics model to demonstrate that a synergistic policy scheme of subsidies, landfill fees, and penalties is beneficial in promoting recycling by introducing a subsidy and penalty mechanism. With the further development of research and practice, more scholars have conducted a more systematic study of drivers by constructing analytical frameworks and models. Lopez Ruiz et al. [10] constructed an analytical framework based on circular economy theory and obtained that insufficient supply of C&DW, imperfect collection and classification standards, lack of market demand for recycled products, immature recycling technology, low cost of natural aggregates, poor environmental awareness, imperfect regulations and legislation, insufficient supervision by regulatory authorities, lack of incentive policies, and insufficient publicity and education on recycling are the constraints of C&DW recycling. After systematically reviewing the problems of recycling, Kabirifar et al. [11] focused on the factors associated with the recycling process, including the application and monitoring of construction site waste management programs, on-site and off-site sorting techniques, incentives or penalties for contractors, demolition techniques, and carrying out plans as recycling drivers. Liu et al. [12] identified and quantitatively analyzed the KDs of recycling in China with the help of stakeholder theory and grey DEMATEL theory, including laws and regulations, the degree of compulsion of normative standards, environmental awareness, C&DW supply, and sales of recycled products. By reviewing 105 pieces of literature, Zhao [13] summarized 35 drivers, including the perfection of laws and regulations, the supervision of the government and the public, and the attitude of stakeholders.

### 2.2. Literature on C&DW Recycling Collaborative Governance Strategy

Multisubject collaborative governance refers to the act of optimizing structure, coordinating interests, and deeply integrating knowledge and resources among multiple subjects in order to obtain complementary advantages and the nonlinear utility of system superposition [14]. The government is the first responsible subject and should play a leading role in the recycling process. It is also a consensus among scholars that owners, contractors, and recycling companies, which are at the supply and demand ends of the C&DW reverse supply chain, should also play an important role in the supply chain [15, 16]. Liu et al. [17] pointed out that government plays an important role in the decision-making of recycling companies, explored the impact of two recycling capacity expansion strategies on profits and the environment, and suggested that despite their conflicting goals in recycling, both government and recycling companies tend to choose the same strategy when recycling handling capacity is low. Tilaye and van Dijk [18] stated that contractors can meet owners' requirements for recycling governance by providing and following an on-site management plan that specifically includes a clear estimate of C&DW and a comprehensive plan for collection classification. Liu et al. [12] proposed that recycling enterprises in the industry chain cannot rely on government subsidies alone to reduce costs, they should form a synergistic linkage with more responsible subjects upstream and downstream of the industry chain to create a new industry chain development mode. Other scholars have studied the game relationship among the government, contractors, and recycling firms, revealing the underlying mechanisms of the strategic choices of the three parties. Their findings contribute to the understanding of the behaviors, demands, and the role of collaborative governance of resource utilization stakeholders [19, 20].

### 2.3. Knowledge Gap

Existing studies on recycling drivers and multisubject collaborative governance have been conducted at some depth, but there lacks a systematic study on multiple and complex relationships between subjects and drivers, and fail to clearly reveal the best way for subjects to collaboratively govern C&DW and how to do so. The distinctive features of new district development make the related research of recycling different from general areas. Therefore, the knowledge gap can be further determined.

1. Few studies have analyzed KDs for the recycling of the new district development. The new district development recycling governance is a more demanding and complex process. Therefore, attention to its KDs is essential to determine the best way of collaborative governance to promote efficient recycling in the new district development.
2. A social network-based perspective would be more useful than other approaches. How to construct an analytical model that can analyze the relationship not only between drivers, but also between governance subjects and between governance subjects and drivers, and explore the ways of these interdependencies and how to adopt appropriate governance strategies to reach the new district development recycling goals is a problem to be solved.

## 3. Methodology

Social networks are classified into unimodal and bimodal networks based on the characteristics of the set of actors and the properties of the connections between them. A bimodal network indicates that the network under the study is bimodal, i.e., it includes a metric for two sets of actors or a set of actors and a set of events [21]. The development of C&DW in the new district involves multiple governance subjects and requires a variety of drivers to work together in a complex social network environment, and the relationship network formed by various drivers with the interaction of subjects is a 2-mode social network. The network can present the collaborative relationship between subjects through KDs jointly promoted or influenced by subjects. Based on this, this paper adopts a 2-mode social network for subject-driver relationship analysis and a 1-mode social network for the relationship analysis within the governing subjects and between drivers. The specific steps and methods are as follows:

**Step 1 .**

Identifying the drivers and related governing subjects of the new district recycling.

Although there are some differences in the composition and drivers of new district development recycling in countries with different systems, socioeconomic cultures, and natural environmental conditions, the basic recycling process is generally the same. It is possible to first analyze the recycling process and the governance subjects and basic relationships involved in each stage, as shown in Figure 1. The initial list is constructed by categorizing and organizing the composition of governance subjects and drivers analyzed from the literature, then revised and supplemented by a semistructured questionnaire survey of several comparable new districts to identify recycling governance subjects and drivers.

**Step 2 .**

Constructing a recycling governance subject-driver adjacency matrix.

Based on the identified governance subjects and drivers, a subject-driver relationship questionnaire is developed for the assessment of the relationship between governance subjects and drivers, and the questionnaire is designed in the form of a structured matrix. In order to minimize the influence of the subjective preferences of the dominant participants, and considering that the judging requires more specialized theoretical knowledge and the number of relationships to be judged is large, the questionnaire survey should not be conducted by distributing a large number of questionnaires, and the Delphi method is appropriate for judging relationships. The relationship is assessed using a five-point Likert scale, with “7” indicating very strong influence, “5” indicating influence, “3” indicating average influence, “1” indicating very little influence, and “0” indicating no influence. After obtaining the questionnaire data, the subject-driver adjacency matrix is constructed. The criteria for determining the relationship between the nodes of the adjacency matrix are as follows: ① when the total number of people choosing “7” and “5” is greater than half of the number of researchers, it means that the subject has influence on drivers, and the relationship value in the matrix is set to 1. ② When the total number of people choosing “0” and “1” is greater than half of the research population, it means that the subject has no influence on drivers, and the relationship value is set to 0. If there are situations other than ① and ② in the final research data, a second round of survey will be set for the specific question data.

**Step 3 .**

Constructing a 2-mode social network model.

The subject-driver adjacency matrix is substituted with UCINET software for model visualization, and four metrics of the 2-mode social network are analyzed: degree centrality, mediator centrality, proximity centrality, and core-periphery analysis. Degree centrality reflects the centrality of nodes, the higher the degree centrality, the higher the associated points and the more important the position in the network; the intermediary centrality reflects the interrelationship between two nonadjacent nodes in the network and the degree of dependence on other nodes in the network; the proximity centrality indicates the proximity of actors to other actors in the network; and the core-periphery structure is an ideal structural pattern that divides both rows and columns into two categories, with subjects and elements closely related in the core part and more sparsely related in the edge part.

**Step 4 .**

Proposing a new district development and recycling the collaborative governance strategy.

Based on the analysis results and connotations of collaborative governance from the 2-mode social network and the two 1-mode social networks, the collaborative governance strategy is systematically proposed in two dimensions: subject-organizational collaboration and resource collaboration. Organizational collaboration is mainly reflected in the positioning of roles, power and responsibility, benefit and risk distribution among governance subjects in the whole process of recycling, which is the external reflection of various related relationships formed by mutual cooperation among different governance subjects and is the basis of the composition of the governance system. Resource collaboration is the integration and interaction of tangible and intangible resources among governance subjects and is the guarantee of the operation of the governance system. Organizational and resource collaboration is coupled through interactive relationships and mutual support, which work together to ensure the achievement of dynamic collaborative governance goals in economic, ecological, and social contexts during different development periods of the new area.

## 4. 2-Mode Network Model Construction

### 4.1. Network Node Determination

Based on the establishment time, scale, and development stage of 19 national-level new districts in China, Chongqing Liangjiang New District, Guizhou Gui'an New District, Dalian Jinpu New District, Sichuan Tianfu New District, and Nanjing Jiangbei New District, which have certain comparability, are selected as the research's new subjects. The semistructured questionnaire analysis of the new research area is used to determine the governance subjects and drivers. The respondents to the questionnaire are mainly the government, owners, contractors (including demolition companies), transportation companies, recycling companies, and other related management personnel. A total of 60 semistructured questionnaires were filled out independently by relevant management personnel in the five research areas after the symposium with our research team to guarantee the questionnaire quality. After statistical analysis of the questionnaire, eight types of governance subjects, government (S1), owners (S2), contractors and or demolition companies (S3), recycling companies (S4), transportation companies (S5), related R&D units (S6), financial institutions (S7), and the public and media (S8), are identified as the subject nodes in the 2-mode network. 29 recycling drivers are event nodes in the 2-mode network, as shown in Table 1.

### 4.2. Modeling Data Acquisition

The subject-driver relationship questionnaire is designed as a structured matrix to assess the relationship between subjects and drivers in Nanjing Jiangbei New District. According to the set of questionnaires, 2 rounds of survey interviews were conducted. In order to improve the reliability and representability of the results, a total of 48 experts were interviewed, all of them are management personnel who have engaged in or plan to engage in the work related to the new district recycling and experts, scholars, the media, and the public who know more about the new district, as shown in the following table.

## 5. Results and Discussion

### 5.1. 2-Mode Network Visualization and Data Analysis

The recycling subject-driver network consists of 8 governing subjects and 29 drivers, connected by 136 links. The red circles represent the governing subjects, and the blue squares represent the drivers. The links between subjects and drivers refer to the subjects' ability to handle, control, and drive the drivers. The visualization model is shown in Figure 2.

The original 2-mode network is converted into a 1-mode network of governing subjects (Figure 3) and a 1-mode network of drivers (Figure 4). In the subject-subject network shown in Figure 3, each node represents a type of subject, and each link represents the number of drivers that neighboring subjects can handle and promote together; the greater the number, the wider the width of the link lines presented in the network. In the driver-driver network shown in Figure 4, each node represents a kind of driver, while each link represents a relationship between drivers. The two 1-mode networks allow a clearer view of the key governing subjects and the KDs, and the strength of these interrelationships can be quantified.

#### 5.1.1. Centrality Analysis

Degree centrality, intermediary centrality, and proximity centrality metrics are examined in conjunction with the recycling subject-driver network.

*(1) Subject Centrality*. The results of the subject centrality analysis are shown in Table 3. The table shows that S1 (government) has the highest centrality because it has the influence to deal with the majority of drivers. S2 (owners), S3 (contractors), and S5 (recycling companies) are ranked second, third, and fourth, respectively, and the three are defined as core supply chain subjects in this paper. This finding suggests that governments and core supply chain subjects have greater access to resources to control drivers and can generate greater impetus for collaborative governance, while at the same time, they are likely to work with a wider range of subjects. In terms of closeness and centrality, S1 (government) scores the highest, indicating that the government has the shortest path of influence on other subjects, followed by S2 (owners), S3 (contractors), and S5 (recycling companies), indicating that the four subjects are most closely connected to other participating subjects and are in a more central position. Interestingly, the ranking of subjects in terms of degree, intermediation, and closeness centrality is similar. S6 (financial institutions) and S7 (public and media) have low degree centrality, intermediary centrality, and closeness centrality. The main reason may be that these subjects have a low degree of expertise in the governance of recycling in new districts, especially the media and financial institutions. However, their contribution to collaborative recycling governance cannot be ignored. Specifically, the media can play an effective role in monitoring illegal dumping of the construction waste, assessing the strength of government regulation, and promoting benchmark projects, thus leading to macrolevel cooperation among subjects to collectively manage construction waste.

*(2) Driver Centrality*. The results of drivers' centrality calculation are shown in Table 4, and the correlation analysis is as follows:

The factors with the highest degree of centrality are I8 (completeness and rationality of the policy system), I12 (new project review and approval system), followed by I3 (degree of collaboration between demolition and new construction plans), and I13 (tender document requirements for waste disposal), and most subjects must pay attention to these four KDs because they cannot be handled and promoted by only one subject. This shows that in order to achieve collaborative governance, while emphasizing a complete and reasonable incentive and constraint policy by the new regional government, active collaboration and cooperation of all supply chain subjects are needed to create a multisubject collaborative effect. The study also found that the degree centrality of drivers such as I1 (special plan for recycling), I9 (construction, operation, and maintenance of an information platform), I16 (construction site management level), I20 (rationality of resource-based facility construction), and I23 (matching degree of recycled products and new district demand) are also high, indicating that these are also the tasks that collaborative governance should focus on.

The drivers with the highest intermediary centrality are I8 (completeness and rationality of the policy system) and I12 (review and approval system for new projects), followed by I23 (matching degree of recycled products and new district demand) and I3 (degree of collaboration between demolition and new construction plans), which are similar to the elements with the highest degree of centrality. The higher the value of the intermediary centrality of drivers, the higher the number of times they act as a bridge for the shortest influence path between nodes in the network, and the more critical their position in the network. Handling such drivers requires the cooperation and collaboration of more related subjects, and if these factors are not handled well or neglected, they can easily lead to other problems.

The higher the value of intermediary centrality of drivers, the higher the number of times they act as a bridge of the shortest influence paths between nodes in the network, and more critical their position in the network. Handling such drivers requires the cooperation and collaboration of more related subjects, and if these factors are not handled well or neglected, they can easily lead to other problems. For example, if the on-site management level cannot be improved through institutional constraints on the contractor, even if a feasible recycling special plan is formulated, and the coordination of demolition and new construction plans is strengthened, it will not be able to efficiently match the output of recycled products with the demand of the new district. The governance elements with the highest degree and betweenness centrality are I8 (completeness and rationality of the policy system) and I12 (review and approval system for new projects), followed by I3 (degree of collaboration between demolition and new construction plans) and I13 (tender document requirements for waste disposal). These factors are the same as the factors with the highest degree and betweenness centrality, and the factors with high closeness centrality are usually related to key participants and have a huge impact on the network.

#### 5.1.2. Core-Periphery Analysis

In order to further clarify the main subjects and KDs of recycling, this paper conducts the core-periphery analysis of the subject-driver network, and the density matrix is shown in Table 5. The final fit is 0.772, indicating that the governance subject-driver network structure conforms to the ideal core-periphery structure. The density of core to periphery and peripheral to core is 0.648 and 0.404, respectively, which indicates that the core governance subject is strongly correlated with edge drivers, but the connection between the edge governance subject and KDs is relatively loose. Although financial institutions, media, and other governance subjects are closely related to drivers, the network of governance subject-driver presents a core-periphery structure with a high density of connection between cores. Based on this analysis, this paper identifies 4 core governance subjects and 15 KDs.

### 5.2. Discussion

Based on the connotation of collaborative governance and the results of the social network analysis mentioned above, the strategies of collaborative governance are discussed as follows.

#### 5.2.1. Governance Strategy Based on Organizational Collaboration

1. Build a government-enterprise collaborative governance platform, and define the power, responsibility, and obligation of each party based on the interest balance system.
2. From Figure 3, it can be seen that the government can handle the most drivers, followed by owners, contractors, and recycling companies, showing a strong power similarity. This requires the government to maintain a leading position and perform government functions while paying attention to the core subjects of the supply chain, which has a promotion effect on recycling. The government should build a collaborative governance platform to determine and fulfill their respective powers, responsibilities, and obligations in a complete, practical, and reasonable manner based on the balance of interests.
3. Build a benefit and risk distribution mechanism for cooperation and competition among supply chain subjects.
4. Based on the strong similarity of power among owners, contractors, and recycling enterprises as shown in Figure 3, the three are typical cooperative and competitive coexistence relationships. The power and responsibilities should be reasonably divided based on their respective positions and roles in the supply chain, and a win-win benefit and risk distribution mechanism should be constructed.
5. Establish a coordination mechanism for the division of labor among relevant government departments.
6. Based on the fact that I3 (degree of collaboration between demolition and new construction plans) and I2 (functional department's collaborative efforts) are in the top 50% of the ranking KDs, it indicates that the new district government should strengthen departmental linkage, realize information sharing, and establish a sound collaborative work mechanism for the whole process of recycling management.
7. Establish a media-public collaborative participation monitoring mechanism.
8. Based on the fact that the media and public play an important role in advancing the top 50% of KDs, such as I27 (application ratio of recycled products) and I29 (attitude of stakeholders participated in governance), they should also be given the responsibility of social monitoring and promotion.

#### 5.2.2. Governance Strategy Based on Resource Coordination

1. Build a resource collaboration mechanism between the government and supply chain subjects.
2. I8 (completeness and rationality of the policy system) is ranked No. 1 KD, which is closely related to the supply chain subjects; the government should systematically formulate a practical policy system based on the principle of win-win cooperation with relevant subjects on the basis of equal communication, and promote the division of labor and cooperation among supply chain subjects to carry out their work. At the same time, I12 (review and approval system for new projects) can be used as a breakthrough, and I3 (degree of collaboration between demolition and new projects) can be used as a means to ensure that recycling is implemented on the ground in a timely manner, and also to provide conditions to ensure the balance of construction waste supply and demand as much as possible. In order to guarantee the orderly implementation of recycling, the government should also compile a special plan for recycling (I1) and build an information platform (I9) on the basis of full research and extensive consultation, so as to guide the work of supply chain subjects in the new district from the top-level design and realize information sharing and communication between the government and the main subjects of the supply chain. At the same time, the supply chain subjects should also regulate and reasonably allocate their resources according to the requirements of policies and systems, for instance, owners should put forward the requirements for waste disposal in the tender documents according to policies (I13), contractors should manage the construction sites according to system requirements (I16), and recycling enterprises should reasonably build resource recycling facilities according to the recycling special plan (I20).
3. Build a resource collaboration mechanism for the main subjects of the supply chain.
4. I13 (tender documents' requirements for waste disposal) and the application of recycled products in the bidding documents have an interactive relationship with I16 (construction site management level), I18 (C&DW quality), I27 (application ratio of recycled products), I20 (rationality of recycling facility construction), and I23 (matching degree of recycled products and new district demand). Therefore, on the premise of complying with the policy requirements of the new district, owners should conduct sufficient research and in-depth communication with relevant market subjects, and reasonably determine the requirements for construction waste treatment and application of recycled products in the bidding documents based on the principle of win-win cooperation and clarify the matching quotation requirements, payment methods, and division of risk and responsibility. Similarly, the resource application of contractors has an interactive relationship with the resource application of recycling enterprises. Thus, the supply chain subjects should actively participate in I9 (construction, operation, and maintenance of the information platform) and establish a resource collaboration mechanism for supply chain subjects to achieve win-win cooperation through information sharing on the information platform.

## 6. Conclusion

This paper analyzes the complex relationship between the subjects and drivers of recycling governance by using SNA in order to present the necessity of collaboration among multiple subjects and to find collaborative governance strategies. Through literature analysis and field research, 8 governance subjects and 29 drivers of recycling in the new district are identified. The analysis of subject centrality shows that the government has the highest degree of centrality, followed by owners, resource utilization companies, and contractors (including demolition companies), indicating that they have more influence in the collaborative governance of recycling. Factor centrality analysis shows that drivers I8 (completeness and rationality of the policy system) and I12 (review and approval system for new projects) have the highest degree of centrality, followed by I3 (degree of collaboration between demolition and new construction plans), I13 (tender documents' requirements for waste disposal), I1 (special plan for recycling), I9 (construction, operation, and maintenance of the information platform), and I16 (Construction site management level). The core-periphery analysis identifies a total of 4 core subjects and 15 KDs with strong relationships with each other. Finally, this paper proposes a collaborative strategy based on the organization of the subjects and resources under the background that different governing subjects promote and deal with multiple drivers through the analysis of the subject-subject network and driver-driver network.

As a fundamental study on collaborative governance of recycling, this paper elucidates the complex relationship between governance subjects and drivers more systematically than previous studies by using 2 models of the social network analysis. The research results provide a basis for each subject to clarify the key subjects that need to be collaborated and the KDs that need to be jointly promoted. The proposed synergistic strategy provides a reference for the optimal allocation of responsibilities, rights, and resources of the management subjects, which can promote the development of the collaborative management of new district recycling, and thus realize the efficient recycling of construction waste during the new district development.

## Figures and Tables

**Figure 1:** C&DW recycling process, subjects, and basic relationships.

**Figure 2:** Subject-drivers'2-mode network visualization.

**Figure 3:** Subject-subject1-mode network visualization.

**Figure 4:** Driver-driver1-mode network visualization.

**Table 1:** Definitions for the C&DW recycling drivers of new district development.

Drivers	Definition	Source
I1: special plan for recycling	The government's special plan to guide recycling and industrial development based on the characteristics of C&DW from the new district development, regional economic, environmental, and social conditions	Added by questionnaire
I2: functional departments collaboration efforts	Division of responsibilities and collaborative work efforts of all relevant government departments	Added by questionnaire
I3: degree of collaboration between demolition and new construction plans	Collaborative development of a regional acquisition, demolition, and new construction plan to facilitate the “local absorption” of C&DW in the new district development	Added by questionnaire
I4: collection and classification of system perfection	The degree of perfection of government regulations related to C&DW site collection and classification	Liu et al. [12]
I5: on-site inspection efforts for collection and classification	Inspections of C&DW collection and classification at construction sites by government functions	Yang and Song [17]
I6: transportation regulatory legislation perfection degree	The government supervises and manages the perfection of the transport behavior regulations of transport enterprises	Jia et al. [9]
I7: transport route supervision efforts	Government's efforts for regulation of transport companies' transport routes and exposure of violations	Liu et al. [12]
I8: completeness and rationality of the policy system	The completeness and rationality of the government's regulatory, binding, and supportive policies based on the characteristics of the new district development	Liu et al. [12]; Zhao [13]
I9: construction, operation, and maintenance of information platform	Government information, interoperability platform, construction, perfection, and operation and maintenance management status	Added by questionnaire
I10: recycled product standards and specifications	Government standards and norms regulating the production and use of recycled products	Zhang et al. [22]
I11: recycled product information and price release	Government-issued recycled product catalog and prices	Added by questionnaire
I12: review and approval system for new projects	Recycling program preparation and disposal approval system for new projects issued by the government	Added by questionnaire
I13: tender documents requirements for waste disposal	Whether there are clauses in the owners' bidding documents that require the tender documents to submit reasonable waste management plans and costs	Added by questionnaire
I14: adequacy and timeliness of payment for waste disposal	Full and timely waste disposal payment from owners to contractors	Added by questionnaire
I15: optimization of project demolition program	Whether the contractor has selected the demolition plan based on the product demand in the new district market	Added by questionnaire
I16: construction site management level	The ability of contractors to determine the level of waste collection, classification, and reuse based on-site conditions	Yang and Song [17]
I17: construction personnel knowledge and skills	The level of skills and knowledge related to waste collection and classification acquired by contractors' personnel through systematic training	Liu et al. [3]
I18: C&DW quality	The C&DW site utilization value is affected by the characteristics of the dismantled objects, the selection of the dismantling scheme, and the site management. This paper mainly refers to the quality affected by humans	Huang et al. [23]
I19: optimization of transportation route selection	Whether the transportation unit considers the economic and environmental benefits comprehensively when choosing the transportation route	Liu et al. [12]
I20: rationality of recycling facility construction	The rationality of the investment scale and site selection of recycling enterprises, fixed + mobile facility scale selection	Added by questionnaire
I21: application rate of new procedure and technology	Application rate of new procedures and technologies in waste treatment and production of recycled products in recycling enterprises	Liu et al. [12]
I22: percentage of recycled materials	The proportion of recycled materials in recycled products produced by recycling companies	Zhang et al. [22]
I23: matching degree of recycled products and new district demand	Whether the recycling company's production decisions for recycled products are based on the new area's market demand	Added by questionnaire
I24: recycled product quality	The quality of recycled products produced by recycling companies	Su and Si [14]
I25: technology support for resource utilization process	Relevant R&D units to dismantle, sort, resource treatment, recycled products production of the whole process, and support technology research and development status	Akinade et al. [24]
I26: financial support	Financial support from financial institutions for recycling companies and R&D institutions	Lin [25]
I27: application ratio of recycled products	The percentage of construction and contractors using recycled products in new construction projects	Yuan et al. [26]
I28: publicity efforts for recycled products	Government, enterprises, media, and other publicity efforts for recycled products and demonstration projects	Wong [27]
I29: attitude of stakeholders participated in governance	Recycling stakeholders' attitudes and awareness of participation in collaborative governance	Jain et al. [5]; Wong [27]

**Table 2:** Expert composition of valid questionnaires.

Occupation	Number	Weight (%)	Related experiences	Number	Weight (%)
Government administrator	6	12.50	2 years	3	8.82
Project owner	6	12.50	3∼4 years	6	17.65
Contractor (including demolition companies) project manager	6	12.50	5 years	8	23.53
Director of transportation companies	6	12.50	6∼8 years	9	26.47
Recycling enterprise manager	6	12.50	Over 10 years	8	23.53
Financial institution manager	6	12.50			
Head of scientific research institution	6	12.50			
Media and public	6	12.50			

**Table 3:** Governance subject centrality.

Participating subjects	Degree	Closeness	Betweenness
S1	1.000	1.000	0.282
S2	0.862	0.843	0.168
S3	0.793	0.782	0.123
S4	0.448	0.573	0.031
S5	0.724	0.729	0.148
S6	0.138	0.462	0.003
S7	0.207	0.483	0.007
S8	0.517	0.606	0.044

**Table 4:** Influencing factor centrality (ranked top 50%, others omitted).

Governance factors	Degree	Closeness	Betweenness
I1	0.750	0.941	0.008
I2	0.625	0.914	0.005
I3	0.875	0.970	0.018
I8	1.000	1.000	0.036
I9	0.750	0.941	0.008
I12	1.000	1.000	0.036
I13	0.875	0.970	0.018
I16	0.750	0.941	0.008
I18	0.625	0.914	0.005
I19	0.625	0.914	0.005
I20	0.750	0.941	0.013
I21	0.625	0.914	0.004
I23	0.750	0.941	0.019
I27	0.625	0.914	0.004
I29	0.625	0.914	0.005

**Table 5:** Core-periphery distribution of main subjects and drivers.

	I1	I2	I3	I18	I19	I20	I8	I21	I16	I13	I27	I12	I9	I23	I19	I22	I4	I5	I7	I10	I11	I14	I17	I24	I25	I26	I28	I29	I15
S1	1	1	1	1	1	1	1	1	1	1	1	1	1	1	1	1	1	1	1	1	1	1	1	1	1	1	1	1	1
S2	1	1	1	1	1	1	1	1	1	1	1	1	1	1	1	1	1	1	0	1	0	1	1	1	1	0	1	1	0
S3	1	1	1	1	0	0	1	1	1	1	1	1	1	1	0	0	1	1	1	0	0	1	1	1	0	0	1	0	1
S5	1	1	1	1	1	1	1	1	1	1	1	1	1	1	1	1	1	0	0	1	1	0	0	1	1	1	0	1	1

S4	1	1	1	1	1	1	1	0	1	1	0	1	1	0	1	0	0	0	0	0	0	0	0	0	0	0	0	1	0
S6	0	0	0	0	0	0	1	0	0	0	1	1	0	1	0	0	0	0	0	0	0	0	0	0	0	1	0	0	0
S7	0	0	1	0	0	1	1	0	0	1	0	1	0	0	0	0	0	0	1	0	0	0	0	0	0	0	0	0	0
S8	1	0	1	0	1	1	1	1	1	1	1	1	1	1	1	1	0	0	0	1	0	0	0	0	0	0	0	1	0

## Data Availability

No data were used to support the findings of this study.
